The article "Klebsiella pneumoniae invasive syndrome with pneumocephalus and extensive cerebral infarction: Case report" was published in 2024. Journal: Heliyon.

# *Klebsiella pneumoniae* invasive syndrome with pneumocephalus and extensive cerebral infarction: Case report

**DOI:** 10.1016/j.heliyon.2024.e25745

**Published:** 2024-02-08

**Authors:** Liangzhe Wu, Changhong Mo, Yihan Xiong, Yanhui Chen, Meng Jin, Kunning Han, Xuejun Fu

**Affiliations:** a The Second Clinical Medical College, Jinan University, 518020, Shenzhen, China; b Department of Intensive Care Unit, Shenzhen People's Hospital, 518020, Shenzhen, China; c Department of Neurology, Shenzhen People's Hospital, 518020, Shenzhen, China

**Keywords:** *Klebsiella pneumoniae*, Multi-organ infection, Intracranial pneumocephalus

## Abstract

A 54-year-old female with diabetes was admitted with fever and altered consciousness. Laboratory tests revealed venous blood glucose level of 43.79 mmol/L. Computed tomography (CT) scans of the head, chest, and abdomen showed a right-sided pneumothorax, consolidation, and atelectasis in the right lung; a large heterogeneous density lesion with fluid and gas-fluid levels in the liver; and scattered gas shadows in both kidneys, respectively. Blood and puncture fluid cultures indicated infection with *Klebsiella pneumoniae*. Based on the susceptibility profiles of the isolates, imipenem was administered intravenously to treat the infection. On the third day of hospitalization, the patient's condition worsened, with head CT showing an extensive cerebral infarction and multiple gas accumulations in the right cerebral hemisphere, as well as a large-area cerebral infarction in the left parietal and occipital lobes. Ultimately, the patient died of multiple organ dysfunction on the fourth day after initial presentation. Although the *Klebsiella pneumoniae* isolates from the patient showed sensitivity to imipenem, this antibiotic shows poor entry into the central nervous system. The death of the patient indicates that the selection of antibiotics that can cross the blood-brain barrier may be crucial in the outcome of this type of case. Therefore, antibiotics that can penetrate the blood-brain barrier should be selected as soon as possible, and empirical treatment must be initiated immediately after clinical suspicion of invasive *Klebsiella pneumoniae*, even if the diagnosis has not been determined.

## 1 Introduction

*Klebsiella pneumoniae* invasive syndrome commonly occurs in patients with immune deficiencies, such as diabetes, alcohol abuse, malignancies, or chronic obstructive pulmonary disease. Uncontrolled blood sugar levels that lead to diabetic ketoacidosis may also be an important factor in the development of this condition. *Klebsiella pneumoniae* is a gram-negative, rod-shaped bacterium that can ferment glucose to produce acid and gas under anaerobic conditions, leading to gas-forming abscesses [1]. Although cases of *Klebsiella pneumoniae* causing hepatic and urinary tract gas-forming abscesses have been reported, their occurrence in the brain is extremely rare [2]. Therefore, antibiotics that can pass through the blood-brain barrier may not be routinely chosen for treatment. The purpose of presenting this case report is to show that the choice of antibiotic may significantly influence outcomes in patients with *Klebsiella pneumoniae* invasive syndrome.

## 2 Case presentation

A 54-year-old female with non-insulin-dependent diabetes who had not received standardized hypoglycemic treatment before was referred to our hospital because she had experienced two weeks of fever and chills and then exhibited disorder of consciousness for half an hour. Two weeks prior to presentation, the patient developed a fever with 37.5 °C being the highest recorded body temperature. She did not exhibit any other obvious symptoms such as abdominal pain or headache. During this period, the patient did not seek treatment at any medical facility. On the day of admission, the patient fell while walking. At that time, the patient was conscious, but half an hour later, a sudden onset of confusion and unresponsiveness occurred. Therefore, the patient was brought to the hospital by family members for medical care. Physical examination of the patient revealed a dull mental state, slurred speech, equal-sized bilateral pupils with a diameter of approximately 3 mm, a sensitive response to light reflex, absent breath sounds in the right lung, and a heart rate of 112 beats per minute. The laboratory tests showed a C-reactive protein level of 197.02 mg/L, procalcitonin level of 10.60 ng/mL, interleukin-6 level of 360.4 pg/mL, white blood cell count of 22.88 × 10^9^/L, neutrophil ratio of 94.6%, lactate level of 6.01 mmol/L, and venous blood glucose level of 43.79 mmol/L. The initial blood pressure of the patient was 96/65 mmHg; Arterial blood gases was 7.22; PCO2 was 8 mmHg; PaO2 was 77 mmHg; and HCO3- was 11.6 mmol/L. Urine volume was 70–80 mL/h. Urgent computed tomography (CT) scans of the head, chest, and abdomen were performed, and the results showed: 1. No apparent brain abnormalities (Fig. 1A), 2. right pneumothorax with consolidation and atelectasis of the right lung (Fig. 1B); 3. Enormous mixed-density lesions in the liver with fluid gas levels and scattered gas shadows were observed in both kidneys (Fig. 1C and D). Immediate interventions included endotracheal intubation, femoral vein catheterization, closed thoracic drainage, percutaneous drainage of the liver abscess, and empirical treatment with imipenem/cilastatin. Blood culture, liver puncture fluid, and pleural drainage revealed *Klebsiella pneumoniae* infection. The isolates showed similar antimicrobial susceptibility and sensitivity to imipenem. Therefore, imipenem was given intravenously (2 g every 8 hours) by drip to treat the infection. Intravenous insulin reduced blood glucose levels, which were monitored once every 1–2 hours, These readings indicated that blood glucose levels fluctuated between 8 and 15 mol/h. Simultaneously, noradrenaline was continuously pumped to boost blood pressure as it fluctuated between 120 and 160/70–90 mmHg, supplementation potassium ion, cool down, protect liver function and other treatment. On the third day of admission, the patient showed bilateral mydriasis with a diameter of about 4 mm, and all reflexes, including light reflex, disappeared. A CT scan of the head showed that the right frontal, parietal, and occipital lobes and the left parietal and occipital lobes were infarcted with multiple accumulations of gas, the midline structure had moved to the left, and a cerebral hernia was formed (Fig. 2A). A chest CT scan revealed a right pneumothorax and consolidation with subcutaneous emphysema in the right neck and chest (Fig. 2B). An abdominal CT scan showed a reduction in the size of the large mixed-density lesion in the liver compared with previous scans, along with new lesions in both kidneys (Fig. 2C and D). On the fourth day after the initial visit, the patient died of multiple organ dysfunction, and her family declined an autopsy.

**Fig. 1:** Axial CT images: **(A)** No obvious abnormalities in the head; **(B)** Right lung showing pneumothorax with lung consolidation and atelectasis (black arrow); **(C)** Enormous lesion in the liver with fluid-gas levels (white arrow); **(D)** scattered gas in both kidneys (white arrow).

**Fig. 2:** Axial CT images: **(A)** Extensive infarction (black arrow) with multiple gas accumulations (white arrow) and formation of cerebral herniation in the right cerebral hemisphere and left parietal and occipital lobes; **(B)** Right lung showing pneumothorax with lung consolidation and atelectasis, subcutaneous emphysema in the neck and chest (white arrow); **(C)** Decreased size of the enormous lesion in the liver, with retained drainage tube (white arrow); **(D)** Minor hemorrhagic foci in both kidneys (white arrow).

## 3 Discussion

The patient was diagnosed with *Klebsiella pneumoniae* invasive syndrome involving the liver, lungs, kidneys, and brain, along with extensive cerebral infarction and pneumocephalus. Blood, thoracic drainage fluid, and liver drainage fluid were collected for bacterial cultivation. All culture results revealed *Klebsiella pneumoniae* infection, and the antimicrobial susceptibility was similar between the different isolates. The patient's routine urine white blood cell, red blood cell, and protein levels had increased, and nitrite tests were positive, suggesting the possibility of a urinary tract infection; however, urine culture was not performed. Similarly, owing to the rapid progression of infection in the brain, cerebrospinal fluid culture was also not performed. In this case, intracranial gas accumulation, extensive cerebral infarction, and cerebral herniation occurred. The presence of intracranial gas suggests the presence of an intracranial infection. Stroke is one of the main complications of intracranial infection. Since the patient was unable to undergo a cranial magnetic resonance imaging examination, we cannot determine whether the infection caused by *Klebsiella pneumoniae* was infectious vasculitis or if the cerebral infarction was caused by septic emboli resulting from the bacteremia. However, cerebral infarction or pneumocephalus is a serious life-threatening event, and the rapid progression of the patient's condition and the rapid deterioration of the brain were considered to be caused by intracranial infection, large-area cerebral infarction, and intracranial gas accumulation. Although *Klebsiella pneumoniae* is sensitive to imipenem, the drug is limited to the peripheral blood, liver, and other areas, and it has difficulty passing through the blood-brain barrier. We often ignore infections of the central nervous system and focus on existing systemic infections. Because infection of the central nervous system is difficult to detect, it may only attract our attention when serious nervous system symptoms manifest. A key point of our case is that *Klebsiella pneumoniae* isolated from this patient was sensitive to both imipenem and meropenem. We have been empirically using imipenem for treatment since the first day of admission, and based on subsequent drug sensitivity results, the protocol has not changed. If we had initiated early treatment with meropenem, which more easily passes through the blood-brain barrier to combat infection in the central nervous system and treat the intracranial lesions, a different outcome may have occurred. Studies have shown that the delayed initiation of antibiotic treatment in patients with bacterial intracranial infections is closely associated with mortality and adverse outcomes [3]. Therefore, for patients suspected to have *Klebsiella pneumoniae* invasion syndrome, using antibiotics that penetrate the blood-brain barrier may be more beneficial to treat intracranial infection when the results of early drug sensitivity are not available.

## 4 Conclusion

Delayed treatment is usually due to the absence of obvious abnormalities on head imaging before lumbar puncture. Therefore, antibiotics that can penetrate the blood-brain barrier should be selected as soon as possible, and empirical treatment must be initiated immediately after clinical suspicion, even if the diagnosis has not been determined due to a delay in lumbar puncture.

## Funding

This study did not receive any funding.

## Informed consent

Informed consent was obtained from the patients’ relatives for the inclusion of their case in this research article and the publication of the corresponding case report, including any relevant medical images.

## Limitation

Without brain magnetic resonance imaging, angiography, and cerebrospinal fluid detection, intracranial lesions and blood vessels could not be identified. Unfortunately, the patient did not undergo a urine culture; therefore, a definitive diagnosis of kidney infection could not be made.

## Open access

This article is licensed under a Creative Commons Attribution 4.0 International Licence, which permits use, sharing, adaptation, distribution, and reproduction in any medium or format as long as you give appropriate credit to the original author(s) and the source, provide a link to the Creative Commons licence, and indicate whether changes were made. The images or other third-party materials in this article are included in the article's Creative Commons licence, unless indicated otherwise in a credit line to the material. If material is not included in the article's Creative Commons licence and your intended use is not permitted by statutory regulations or exceeds the permitted use, permission will be obtained directly from the copyright holder. To view a copy of this licence, visit http://creativecommons.org/licenses/by/4.0/.

## Data availability statement

Data are included in the article/supplement. Materials/referenced in this article.

## CRediT authorship contribution statement

**Liangzhe Wu:** Writing – review & editing, Writing – original draft, Methodology, Investigation, Formal analysis, Data curation. **Changhong Mo:** Writing – review & editing, Writing – original draft, Investigation, Formal analysis, Data curation. **Yihan Xiong:** Formal analysis, Data curation. **Yanhui Chen:** Data curation. **Meng Jin:** Data curation. **Kunning Han:** Writing – original draft, Funding acquisition. **Xuejun Fu:** Writing – review & editing, Writing – original draft, Funding acquisition.

## Declaration of competing interest

The authors declare that they have no known competing financial interests or personal relationships that could have appeared to influence the work reported in this paper.
